The article "DAT (deacylating autotransporter toxin) from Bordetella parapertussis demyristoylates Gαi GTPases and contributes to cough" was retracted in 2025. Reasons: fabricated or falsified data; an official misconduct investigation; misconduct by an author; unreliable results or conclusions.

# DAT (deacylating autotransporter toxin) from *Bordetella parapertussis* demyristoylates Gα_i_ GTPases and contributes to cough

**DOI:** 10.1073/pnas.2308260120

**Published:** 2023-09-25

**Authors:** Yukihiro Hiramatsu, Takashi Nishida, Natsuko Ota, Yuki Tamaki, Dendi K. Nugraha, Yasuhiko Horiguchi

**Affiliations:** ^a^Department of Molecular Bacteriology, Research Institute for Microbial Diseases, Osaka University, Suita, Osaka 565-0871, Japan; ^b^Center for Infectious Disease Education and Research, Osaka University, Suita, Osaka 565-0871, Japan

**Keywords:** *Bordetella parapertussis*, cough, DAT, demyristoylation, G_i_ GTPases

## Abstract

The pathogenic bacteria *Bordetella pertussis* and *Bordetella parapertussis* cause pertussis (whooping cough) and pertussis-like disease, respectively, both of which are characterized by paroxysmal coughing. We previously reported that pertussis toxin (PTx), which inactivates heterotrimeric GTPases of the G_i_ family through ADP-ribosylation of their α subunits, causes coughing in combination with Vag8 and lipid A in *B. pertussis* infection. In contrast, the mechanism of cough induced by *B. parapertussis*, which produces Vag8 and lipopolysaccharide (LPS) containing lipid A, but not PTx, remained to be elucidated. Here, we show that a toxin we named deacylating autotransporter toxin (DAT) of *B. parapertussis* inactivates heterotrimeric G_i_ GTPases through demyristoylation of their α subunits and contributes to cough production along with Vag8 and LPS. These results indicate that DAT plays a role in *B. parapertussis* infection in place of PTx.

## Significance

We identified a toxin named deacylating autotransporter toxin, DAT, of *Bordetella parapertussis*, a pathogenic bacterium that causes a respiratory disease with severe coughing, pertussis-like disease. DAT inactivates heterotrimeric GTPases of the G_i_ family by a mechanism through demyristoylation of the Gα_i_ subunits and contributes to evoking cough. We previously demonstrated that *Bordetella pertussis*, which is closely related to *B. parapertussis*, evokes coughing in host animals through the action of pertussis toxin. Pertussis toxin ADP-ribosylates and inactivates the G_i_ GTPases; however, it remained unclear why *B. parapertussis*, which does not produce pertussis toxin, causes coughing. The present study elucidated that DAT, inactivating the G_i_ GTPases in a different manner, assumes the role of pertussis toxin in *B. parapertussis* infection.

*Bordetella pertussis* and *Bordetella parapertussis* cause highly contagious respiratory diseases, pertussis (whooping cough), and pertussis-like disease, respectively. These diseases are characterized by severe paroxysmal coughing that persists for several weeks and imposes a significant burden on patients, especially infants. The pertussis-like disease due to *B. parapertussis* is shorter in duration but clinically indistinguishable from the disease due to *B. pertussis* and, therefore, often counted as pertussis. In addition, *B. parapertussis* has been detected at significant rates during pertussis outbreaks (1, 2), indicating that the organism spreads concurrently with *B. pertussis* epidemics. Considering that *B. pertussis* and *B. parapertussis* are genetically closely related and share many virulence factors (3), their pathogenicity and the mechanism of their disease development during infection may be similar. Additionally, these bacteria may similarly produce host coughing with shared causative virulence factors. However, we recently uncovered the mechanism of *B. pertussis*–induced cough, in which pertussis toxin (PTx) produced by *B. pertussis* but not *B. parapertussis* is involved in causing coughing, indicating that the mechanisms of cough production by *B. pertussis* and *B. parapertussis* are not identical (4). In *B. pertussis*–induced cough, PTx, virulence-associated gene 8 (Vag8), and lipooligosaccharide (LOS) of the bacterium cooperatively function to trigger the cough reflex. The lipid A moiety of LOS stimulates the generation of bradykinin (Bdk), a potent inflammatory mediator, through interactions with toll-like receptor 4 (TLR4). Vag8 exacerbates Bdk accumulation by inhibiting C1 esterase inhibitor (C1-Inh), the major negative regulator for Bdk biogenesis. The accumulated Bdk sensitizes the transient receptor potential vanilloid 1 (TRPV1) ion channel, a key regulator to evoke coughing, through G_q_ and G_s_ GTPases. Simultaneously, Bdk stimulates an inhibitory cascade on TRPV1 in a G_i_ GTPase-dependent manner. PTx hypersensitizes TRPV1 by inhibiting the action of G_i_ GTPases. Consequently, pertussis patients cough by normally innocuous stimuli. *B. parapertussis* shares Vag8, which is 97.3% identical to that of *B. pertussis*, as well as lipid A contained in lipopolysaccharide (LPS), but not PTx because of mutations in the promoter region of the *ptx* operon (5). These observations imply that *B. parapertussis* without PTx causes host coughing in a totally different manner from *B. pertussis* or that the bacterium produces another virulence factor hypersensitizing TRPV1 in place of PTx.

The article "DAT (deacylating autotransporter toxin) from Bordetella parapertussis demyristoylates Gαi GTPases and contributes to cough" was retracted in 2025. Reasons: fabricated or falsified data; an official misconduct investigation; misconduct by an author; unreliable results or conclusions.

PTx of *B. pertussis* is an enzyme toxin targeting heterotrimeric GTPases, which consist of G_α_, G_β_, and G_γ_ subunits. The function of GTPases depends on guanine nucleotide exchange on the G_α_ subunit between the active guanosine triphosphate (GTP)- and inactive guanosine diphosphate (GDP)-bound states (6), and the functional characteristics of the GTPases are determined by the G_α_ subunits, which are classified into four main families: Gα_s_, Gα_i_, Gα_q_, and Gα_12_. Among these, PTx ADP-ribosylates members of only Gα_i_ and uncouples the subunits from G protein–coupled receptors (GPCRs), which mediate signals from extracellular ligands to heterotrimeric GTPases. As a result, cells intoxicated with PTx become insensitive to ligands for Gα_i_-coupled GPCRs. In the mechanism of pertussis cough, PTx uncouples Gα_i_ from Bdk B2 receptor (B2R) and abrogates the inhibitory cascade against TRPV1, which triggers uncontrollable coughing.

In the present study, we searched for an unknown factor of *B. parapertussis* that inhibits B2R- or Gα_i_-mediated signal transduction similar to PTx, identifying an autotransporter, BPP0449. This autotransporter, which we designated deacylating autotransporter toxin (DAT), exhibited deacylation activity to demyristoylate Gα_i_. Demyristoylated Gα_i_ lost the ability to interact with adenylate cyclase (AC), the downstream effector, which resulted in the uncoupling of Bdk-mediated TRPV1 inhibition. Our results also showed that DAT, Vag8, and LPS of *B. parapertussis* cooperatively cause coughing in mice, indicating that *B. parapertussis* utilizes DAT instead of PTx to cause paroxysmal coughing in hosts through a similar mechanism as *B. pertussis*.

## Results

### *B. parapertussis* Induces Coughing Similar to *B. pertussis*.

We intranasally inoculated mice with *B. parapertussis* in a manner similar to *B. pertussis* in our previous study (4) and observed that mice coughed approximately 1 wk after inoculation (Fig. 1 *A–C* and Movies S1 and S2). The extent of the cough production did not differ between the bacterial strains isolated from humans (12822, 23054, and CZ8234) and sheep (CZ77). We previously reported that not only living *B. pertussis* but also its bacterial lysates caused coughing in mice (4). Similarly, in the present study, the lysates from *B. parapertussis* caused coughing (Fig. 1*D*). In contrast to *B. pertussis*, the deletion of *ptx* genes in *B. parapertussis* did not affect the ability to induce coughing (Fig. 1*E*). The lysate from a Vag8-deficient mutant (Δ*vag8*) and the lysate from the wild-type (WT) strain with LPS eliminated with polymyxin B exhibited a reduced ability to cause coughing. Conversely, the addition of recombinant Vag8 and purified LPS from *B. parapertussis* to respective lysates restored coughing (Fig. 1 *E* and *F*). We also confirmed that *B. parapertussis* produces functional Vag8, which binds to and inactivates C1-Inh, although the expression levels in *B. parapertussis* were lower than those in *B. pertussis* (*SI Appendix*, Fig. S1 *A–D*). Vag8 and LPS from *B. parapertussis* in combination with PTx from *B. pertussis* caused coughing to the same extent as lysate from WT *B. parapertussis* (Fig. 1*G*). These results suggest that Vag8 and LPS of *B. parapertussis* may contribute to cough production; however, *B. parapertussis* does not produce PTx.

The article "DAT (deacylating autotransporter toxin) from Bordetella parapertussis demyristoylates Gαi GTPases and contributes to cough" was retracted in 2025. Reasons: fabricated or falsified data; an official misconduct investigation; misconduct by an author; unreliable results or conclusions.

**Fig. 1.** *B. parapertussis*–induced coughing in mice. (*A*–*C*) Cough production in mice inoculated with *B. parapertussis* (Bpp) strains 12822, 23054, CN8234, and CZ77. The number of coughs was counted for 5 min per day for 11 d from days 4 to 14 postinoculation (*A*), and the total number is shown (*B*). The number of bacteria recovered from the tracheas and lungs was counted on day 14 (*C*). (*D*–*H*) Cough production in mice inoculated with bacterial lysates and components of *B. parapertussis*. WT (*D*–*H*), *Tlr4*^−/−^ (*H*), and *Kng1*^−/−^ (*H*) mice were inoculated with various preparations of bacterial components on days 0 to 4 (arrows in panel *D*). The inoculated preparations were as follows: bacterial lysates of *B. parapertussis* 12822 WT (*D*–*H*), Δ*ptx* (*E*), and Δ*vag8* (*E*); bacterial lysate of *B. parapertussis* 12822 WT that was pretreated with Detoxi-Gel (polymyxin B [Polmx +]) (*F*); Vag8 (*E* and *G*) and LPS (*F* and *G*) from *B. parapertussis* 12822; and PTx from *B. pertussis* 18323 (*G*). The number of coughs was counted for 5 min per day from days 4 to 14 (*D*) and is expressed as the sum of coughs for 11 d (*E*–*H*). (*I*) Effects of antagonists on *B. parapertussis*–induced coughing. Mice were inoculated with antagonists against B1R, B2R, TRPV1, and TRPA1, or Dulbecco's modified phosphate-buffered saline (PBS) (300 µL) prior to inoculation with bacterial lysate of *B. parapertussis* 12822. The sum of coughs from days 4 to 14 is shown. (*J*) Bdk concentrations in the BALF of mice inoculated with bacterial lysate of *B. parapertussis* 12822. The concentrations of Bdk were determined on day 4 by ELISA. SS medium without bacteria (*A*–*C*) or PBS (*D*–*J*) was used for mock inoculation. Each plot represents the mean and SEM (*A* and *D*). Each horizontal bar represents the mean and SEM (*B*, *E*–*J*) or the geometric mean and geometric SD (*C*). Data were obtained from two independent experiments (n = 8) and statistically analyzed by one- (*B*, *E*–*G*, and *I*) or two- (*H*) way ANOVA with Tukey’s multiple-comparison test or the unpaired *t* test (*J*). *P < 0.05, **P < 0.01, ***P < 0.001, and ****P < 0.0001.

As mentioned described above, our previous study demonstrated that *B. pertussis* causes coughing in host animals by stimulating the TLR4–Bdk–B2R–TRPV1 pathway (4). Therefore, we examined whether *B. parapertussis* causes coughing similar to *B. pertussis* (*SI Appendix*, Fig. S2). Lysate from *B. parapertussis* caused less frequent coughing in TLR4-deficient mice than WT mice (Fig. 1*H*). Similar results were obtained in high-molecular-weight kininogen (HK)-deficient (*Kng1*^−/−^) mice, which do not produce Bdk because of the lack of its precursor, HK. Mice preadministrated with antagonists against B2R and TRPV1, but not B1R and TRPA1, exhibited reduced levels of coughing in response to lysate from *B. parapertussis* (Fig. 1*I*). Bdk concentrations in the bronchoalveolar lavage fluid (BALF) of mice increased 4 d after intranasal inoculation of the bacterial lysate (Fig. 1*J*). These results indicate that *B. parapertussis*, as well as *B. pertussis*, stimulates the TLR4–Bdk–B2R–TRPV1 pathway to cause coughing.

The article "DAT (deacylating autotransporter toxin) from Bordetella parapertussis demyristoylates Gαi GTPases and contributes to cough" was retracted in 2025. Reasons: fabricated or falsified data; an official misconduct investigation; misconduct by an author; unreliable results or conclusions.

### Identification of DAT As a Causative Agent for Cough Production.

*B. parapertussis* likely stimulates the TLR4–Bdk–B2R–TRPV1 pathway via the action of LPS and Vag8 similar to *B. pertussis*; however, *B. parapertussis* does not produce PTx, which is essential for *B. pertussis* to evoke coughing. In the *B. pertussis*–induced coughing, LOS and Vag8 stimulate and increase Bdk generation. Bdk stimulates the phosphorylation and sensitization of TPRV1 through B2R, which is coupled with G_q/11_, G_i_, and G_s_ GTPases (4, 7, 8). PTx inactivates G_i_ GTPases, which transduce a downstream inhibitory signal from B2R, and exacerbates the Bdk-induced sensitization of TRPV1 by increasing intracellular cyclic adenosine monophosphate (cAMP) (*SI Appendix*, Fig. S2). To explore whether *B. parapertussis* produces a virulence factor(s) functionally corresponding to PTx, we examined its ability to inactivate G_i_ GTPases. To this end, we determined the intracellular concentration of cAMP in T98G human glioblastoma cells treated with Bdk, which stimulates and inhibits cAMP production through G_s_- and G_i_-mediated pathways, respectively (7, 8). If *B. parapertussis* inactivates G_i_ GTPases, it should increase cAMP accumulation upon Bdk treatment in this experimental system. A *B. parapertussis* mutant deficient in adenylate cyclase toxin (Δ*cyaA*) was used in this assay because CyaA per se increases intracellular cAMP (9). The living Δ*cyaA* mutant and its lysate and culture supernatant increased cAMP in the presence of Bdk, similar to PTx, indicating the inactivation of B2R-coupled G_i_ GTPases (Fig. 2*A*). *Bordetella* species, including *B. parapertussis*, exhibit two distinct phenotypic phases, Bvg^+^ and Bvg^−^, which are regulated by the BvgAS two-component system in response to environmental alterations (9). At 37 °C in standard *Bordetella* media, the BvgAS system promotes the transcription of a set of virulence factors, including CyaA and PTx. Conversely, this system is inactivated in the presence of MgSO_4_ and nicotinic acid, and the bacteria shut down the expression of the virulence factors. The Bvg^+^ phase is generally considered to represent the virulent phenotype, while Bvg^−^ phase represents the avirulent phenotype. The Bvg^−^-locked mutant of *B. parapertussis*, which constitutively exhibits the Bvg^−^ phenotype (10, 11), did not increase Bdk-induced cAMP production (Fig. 2*A*). These results indicate that *B. parapertussis* produces a virulence factor(s) that inactivates G_i_ GTPases in a BvgAS-dependent manner. We then fractionated the culture supernatant of Δ*cyaA* by anion exchange chromatography, examined the fractions for the ability to increase cAMP in the presence of Bdk, and identified by mass spectrometry four proteins (BPP0449, BPP3876, PrlC, and SphB3) contained only in fractions #12–16 that enhanced Bdk-induced cAMP production (Fig. 2*B* and *SI Appendix*, Table S1). Among the four proteins, the deletion of *bpp0449*, but not *bpp3876*, *sphB3*, or *prlC*, abolished the ability of the bacterial culture supernatant to enhance Bdk-induced cAMP production (Fig. 2*C*). When Δ*bpp0449*Δ*cyaA* was complemented with a BPP0449-expressing plasmid, p*bpp0449*, the bacterial enhancing ability was restored (Fig. 2*D*). Immunoblotting analyses detected BPP0449 in bacterial lysates and culture supernatants from different *B. parapertussis* strains under Bvg^+^ phase conditions (*SI Appendix*, Fig. S3 *A* and *B*), indicating that BPP0449 is generally produced by *B. parapertussis* in the Bvg^+^ phase. Orthologues of *bpp0449* in *B. pertussis* were not found by a BLAST search (https://blast.ncbi.nlm.nih.gov/Blast.cgi). The *bpp0449* gene encodes an autotransporter protein. Hereafter, based on the following results, we refer to BPP0449 as deacylating autotransporter toxin, DAT.

The article "DAT (deacylating autotransporter toxin) from Bordetella parapertussis demyristoylates Gαi GTPases and contributes to cough" was retracted in 2025. Reasons: fabricated or falsified data; an official misconduct investigation; misconduct by an author; unreliable results or conclusions.

**Fig. 2.** Identification of BPP0449 causing Bdk-dependent accumulation of intracellular cAMP. (*A*–*D*) Increase in Bdk-induced cAMP production in T98G cells incubated with *B. parapertussis* preparations. T98G cells were incubated with PTx (10 ng/mL) (*A*), *B. parapertussis* 12822 mutant strains (MOI 1) (*A*), and bacterial lysates (100 µg/mL) (*A*) or 100-fold diluted culture supernatants (*A*, *C*, and *D*) of the bacteria for 24 h. Hank’s-HEPES BSA was used for mock treatment. The bacterial culture supernatant of *B. parapertussis* 12822-Δ*cyaA* was subjected to anion exchange chromatography, and the absorbed proteins were eluted with a linear gradient of NaCl from 0 to 0.5 M. The eluted fractions (no. 1 to 25), Mock (20 mM Tris-HCl, pH 8.0), the culture supernatant, and a flow-through fraction (FT) were diluted 100-fold in Hank’s-HEPES BSA and applied to T98G cells (*B*). The cells were then treated with 100 nM Bdk for 30 min, and intracellular cAMP was measured by ELISA. Each bar represents the mean and SEM (*A*, *C*, and *D*, n = 6; *B*, n = 3). Data were obtained from one (*B*) or two (*A*, *C*, and *D*) independent experiments and statistically analyzed by one-way ANOVA with Tukey’s multiple-comparison test (*B*) or two-way ANOVA with the Sidak multiple-comparison test (*A*, *C*, and *D*). ****P < 0.0001.

DAT is one of the autotransporter proteins consisting of passenger and translocator domains (Fig. 3*A*). After being transported into the periplasm via a signal peptide, the passenger domain of autotransporter proteins is translocated across the outer membrane through a conduit formed by the translocator domain. Some autotransporter proteins undergo proteolytic cleavage between the passenger domain and the translocator domain, and the former is liberated into the extracellular milieu (12). We generated recombinant proteins covering the passenger domains of DAT and BatB (13), an autotransporter protein encoded by *bpp0452*, the amino acid sequence of which is 48.6% identical to that of DAT from *B. parapertussis* (Fig. 3*A*), and examined the two proteins for the enhancement of Bdk-induced cAMP production. We used BatB, which is most homologous to DAT in *B. parapertussis*, as a negative control. When extracellularly added, DAT, but not BatB, augmented the Bdk-induced cAMP production in the cells (Fig. 3*B*). In mouse coughing experiments, bacterial lysates from Δ*dat* did not cause coughing, but Δ*dat* lysate complemented with DAT caused coughing to the same extent as the WT lysate (Fig. 3*C*). Inoculation of DAT in combination with LPS and Vag8, but not DAT alone, caused coughing (Fig. 3*D*), indicating that DAT plays a role in cough induction similar to PTx of *B. pertussis*.

**Fig. 3.** Involvement of DAT in *B. parapertussis*–induced coughing. (*A*) Schematic representations of DAT and BatB. The domains of DAT and BatB were analyzed using SignalP 6.0 (14) and Pfam 35.0 (15). HAT-tagged recombinant proteins covering the passenger domain of DAT and BatB were constructed from the amino acid residues 42 to 1251 and 43 to 1413, respectively. (*B*) Increase in Bdk-induced cAMP production in T98G cells incubated with DAT. T98G cells were incubated with 100-fold diluted culture supernatant of *B. parapertussis* 12822-Δ*cyaA* and the indicated concentrations of DAT or BatB for 24 h. Hank’s-HEPES BSA was used for mock treatment. The cells were then treated with 100 nM Bdk for 30 min, and intracellular cAMP was measured by ELISA. Each bar represents the mean and SEM (n = 6). (*C* and *D*) Cough production in mice inoculated with bacterial lysates and components of *B. parapertussis*. Mice were inoculated with bacterial lysates of *B. parapertussis* 12822 WT or Δ*dat* strains and LPS, Vag8, and/or DAT from *B. parapertussis* 12822. The sum of coughs from days 4 to 14 is shown. Each horizontal bar represents the mean and SEM (n = 8). Data were obtained from two independent experiments and statistically analyzed by two-way ANOVA with the Sidak multiple-comparison test (*B*) or one-way ANOVA with Tukey’s multiple-comparison test (*C* and *D*). **P < 0.01, ****P < 0.0001.

The article "DAT (deacylating autotransporter toxin) from Bordetella parapertussis demyristoylates Gαi GTPases and contributes to cough" was retracted in 2025. Reasons: fabricated or falsified data; an official misconduct investigation; misconduct by an author; unreliable results or conclusions.

### DAT Inactivates Gα_i/o/z_ GTPases by Deacylating Activity.

We then explored the mechanism underlying the DAT-induced inactivation of G_i_ GTPases. We generated T98G cells stably expressing DAT, BatB, and PTx S1, a catalytic subunit of PTx, and found that the intracellular expression of DAT, but not BatB, enhances Bdk-induced cAMP production, similar to that of PTx S1 (Fig. 4*A*). These results suggest that DAT intracellularly functions to inactivate G_i_ GTPases. A PROSITE search (https://prosite.expasy.org/prosite.html) revealed that DAT, but not BatB, contains a GDSL lipolytic enzyme motif ([LIVMFYAG](4)-G-D-S-[LIVM]-x(1, 2)-[TAG]-G), of which Ser serves as the catalytic residue (16, 17) (Fig. 4*B*). DAT exhibited deacylating activity against artificial substrates, including *p*-nitrophenyl (pNP)-butyrate, -myristate, and -palmitate, which form chromatic *p*-nitrophenol upon removal of the fatty acid groups (Fig. 4*C*). In contrast, a mutant of DAT, DAT_S571A_, in which the putative catalytic serine residue at amino acid position 571 was substituted with alanine, did not show enzyme activity (Fig. 4 *B* and *D*). Consistently, DAT_S571A_ did not influence Bdk-induced cAMP production (Fig. 4*D*). Additionally, neither bacterial lysates from a *B. parapertussis* mutant producing DAT_S571A_ (*dat*_S571A_) nor purified DAT_S571A_ combined with LPS and Vag8 caused coughing (Fig. 4*E*). These results indicate that DAT inactivates G_i_ GTPases and contributes to cough production through its intrinsic deacylating activity.

**Fig. 4.** Deacylating activity of DAT is essential to cause coughing. (*A*) Increase in Bdk-induced cAMP production in T98G cells expressing *dat*, *batB*, and *ptxA*. After treatment with 100 nM Bdk for 30 min, intracellular cAMP was measured by ELISA. Each bar represents the mean and SEM (n = 6). (*B*) Partial sequence alignment of DAT, BatB, and four representative lipolytic enzymes (GcaT, PlaA, TesA, and SseJ) from *A. salmonicida*, *L. pneumophila*, *E. coli*, and *S.* Typhimurium. All proteins other except BatB contain the GDSL motif. The serine residue required for enzyme activity is shown in red. DAT_S571A_ contains a serine-to-alanine substitution at amino acid position 571 in DAT. (*C*) Deacylating activity of DAT. DAT, DAT_S571A_, and BatB (5 µg/mL) were incubated with 3.25 mM pNP-butyrate, -myristate, or -palmitate in a 96-well plate at 37 °C. The OD_405_ value of each well was measured every minute for 30 min. Each plot represents the mean and SEM (n = 6). (*D*) Increase in Bdk-induced cAMP production in T98G cells incubated with DAT. T98G cells were incubated with the indicated concentrations of DAT or DAT_S571A_ for 24 h and then treated with 100 nM Bdk for 30 min. Intracellular cAMP was measured by ELISA. Each bar represents the mean and SEM (n = 6). (*E*) Cough production in mice inoculated with bacterial lysates and components of *B. parapertussis*. Mice were inoculated with bacterial lysates of *B. parapertussis* 12822 WT or *dat*_S571A_ strains and LPS, Vag8, and DAT or DAT_S571A_ from *B. parapertussis* 12822. The sum of coughs from days 4 to 14 is shown. Each horizontal bar represents the mean and SEM (n = 8). Data were obtained from two independent experiments and statistically analyzed by two-way ANOVA with the Sidak multiple-comparison test (*A* and *D*) or one-way ANOVA with Tukey’s multiple-comparison test (*E*). ****P < 0.0001.

The article "DAT (deacylating autotransporter toxin) from Bordetella parapertussis demyristoylates Gαi GTPases and contributes to cough" was retracted in 2025. Reasons: fabricated or falsified data; an official misconduct investigation; misconduct by an author; unreliable results or conclusions.

The α subunits of the G_i_ family, including Gα_i_, Gα_o_, and Gα_z_, are myristoylated and palmitoylated on the N-terminal glycine and cysteine residues, respectively (Fig. 5*A*). Since DAT, which inactivated G_i_ GTPases, showed deacylating activity against pNP-myristate and -palmitate (Fig. 4*C*), we utilized the click-chemistry-based assay, a reliable method to detect acylated proteins (18, 19) and examined whether it targets acylated Gα_i_. In this assay, T98G cells were treated with myristic acid- or palmitic acid-alkyne, and then, the cell lysates were incubated with biotin-azide, leading to attachment of biotin to the myristoyl and palmitoyl groups through copper-catalyzed alkyne-azide cycloaddition reaction. Subsequent immunoblotting for biotin detected the myristoylated and palmitoylated proteins. The overall profiles of the myristoylated and palmitoylated proteins in T98G cells were largely unaffected by treatment of the cells with DAT (*SI Appendix*, Fig. S4*A*). Myristoylated Gα_i1_ was detected by the combination of the click-chemistry-based assay and anti-HA tag immunoprecipitation with T98G cells expressing functional Gα_i1_ with the HA tag inserted between amino acid positions 91 and 92 (20, 21). The level of myristoylated Gα_i1_ was reduced with time in the cells treated with DAT (Fig. 5*B*). Palmitoylated Gα_i1_ was not detected by our method, probably because palmitoylation of the G_α_ subunits is reversible (22) (*SI Appendix*, Fig. S4*B*). In addition to Gα_i_, Gα_o1_ and Gα_z_ were also demyristoylated by DAT (Fig. 5*C*). As expected, DAT_S571A_ did not demyristoylate the G_α_ subunits (Fig. 5*C* and *SI Appendix*, Fig. S4*B*). We examined whether DAT directly demyristoylates the G_α_ subunits by treating the lysate of *Escherichia coli* coexpressing Gα_i1_ and *N*-myristoyltransferase (NMT) (23) with DAT in the absence or presence of the Gβ_1_γ_2_ subunits. The myristoylation of recombinant Gα_i1_ in *E. coli* was confirmed by the click chemistry-based assay. DAT demyristoyated recombinant Gα_i1_ in the presence of Gβ_1_γ_2_ (Fig. 5*D*). In contrast, DAT did not affect the myristoylation of recombinant Gα_i1_ without the βγ subunits regardless of the presence of GTPγS or GDPβS (*SI Appendix*, Fig. S4*C*), indicating that monomeric Gα_i1_ does not serve as a substrate for DAT in both the active GTP- and inactive GDP-bound states. These results indicate that DAT targets α subunits of the G_i_ family in the heterotrimeric state, similar to the ADP-ribosylating action of PTx (24).

The article "DAT (deacylating autotransporter toxin) from Bordetella parapertussis demyristoylates Gαi GTPases and contributes to cough" was retracted in 2025. Reasons: fabricated or falsified data; an official misconduct investigation; misconduct by an author; unreliable results or conclusions.

**Fig. 5.** Inactivation of G_i_ GTPases by DAT-induced demyristoylation of Gα_i_. (*A*) Sequence alignment of the N-terminal region of the human G_α_ subunits of the G_s_, G_i_, G_q_, and G_12_ families. The α subunits of the G_i_ family contain the myristoylation motif (GXXXS) shown in red. The underlined cysteine residues are putatively palmitoylated. (*B* and *C*) DAT-induced demyristoylation of Gα_i/o/z_ in T98G cells analyzed by the click-chemistry-based assay (18, 19). T98G cells were transfected with expression vectors for HA-tagged Gα_i1_ (*B* and *C*), Gα_o1_ (*C*), or Gα_z_ (*C*) in the presence of myristic acid-alkyne for 24 h and further incubated with 100 ng/mL DAT for the indicated periods (*B*) or 1, 10, and 100 ng/mL (*C*) DAT or 100 ng/mL DAT_S571A_ for 24 h (*C*). Myristoylated G_α_ proteins (myr-Gα_i1_, -Gα_o1_, and -Gα_z_) were detected by immunoblotting with anti-biotin antibody as described in *SI Appendix*, *Materials and Methods*. Gα_i1_ (*B* and *C*), Gα_o1_ (*C*), and Gα_z_ (*C*) were independently detected with antibodies against each protein as internal controls. The blot images are representatives of two independent experiments. The band intensities of myr-Gα_i1_, -Gα_o1_, and -Gα_z_ were measured using Fiji software (25) and are presented as a ratio relative to those of Gα_i1_, Gα_o1_, and Gα_z_, respectively. (*D*) DAT-induced demyristoylation of recombinant Gα_i_. Bacterial lysates from *E. coli* strain coexpressing Gα_i1_ and NMT were treated with GDPβS for 1 h and then further incubated with 0.1, 1, and 10 µg/mL DAT or 10 µg/mL DAT_S571A_ in the absence or presence of Gβ_1_γ_2_ for 2 h. The amount of myr-Gα_i1_ was calculated as described above. The blot images are representatives of two independent experiments. (*E*) Interactions between Gα_i1_ and AC5 analyzed by a FRET assay. T98G cells were transfected with Gα_i1_-CFP and YFP-AC5 expression vectors and then incubated with 100 ng/mL DAT or DAT_S571A_ for 24 h. After treatment with or without clonidine for 30 min, the fluorescence intensities of CFP and YFP were measured, and ΔF_CFP_ and ΔF_YFP_ were calculated as described in *SI Appendix*, *Materials and Methods*. Each bar represents the mean and SEM (n = 6). Note that when FRET occurs between Gα_i1_ and AC5, ΔF_CFP_ and ΔF_YFP_ decrease and increase, respectively. Data were obtained from two independent experiments and statistically analyzed by two-way ANOVA with the Sidak multiple-comparison test. *P < 0.05 and ****P < 0.0001.

The article "DAT (deacylating autotransporter toxin) from Bordetella parapertussis demyristoylates Gαi GTPases and contributes to cough" was retracted in 2025. Reasons: fabricated or falsified data; an official misconduct investigation; misconduct by an author; unreliable results or conclusions.

The myristoylation of Gα_i_ is crucial for interactions with AC, the downstream effector (26, 27). The activity of AC, which catalyzes cAMP production from adenosine triphosphate (ATP), is inhibited by Gα_i_ through the interaction between Gα_i_ and AC (26–28). If DAT inactivates G_i_ GTPases, the interaction between Gα_i_ and AC should not be observed even when the α subunits of the G_i_ family are activated by G_i_-coupled GPCRs. We, therefore, examined the interaction of Gα_i1_ treated with DAT and the AC5 isoform of ACs (29) by a fluorescence resonance energy transfer (FRET)-based assay using T98G cells expressing Gα_i1_-cyan fluorescent protein (CFP) and yellow fluorescent protein (YFP)-AC5, in which interactions between Gα_i1_ and AC5 are detected by a decrease in CFP fluorescence (ΔF_CFP_) and an increase in YFP fluorescence (ΔF_YFP_) because the emission of CFP is used for the excitation of YFP (20). In addition, we used clonidine, an agonist for G_i_-coupled α_2_-adrenergic receptor (30), stimulation of which has been reported to induce the interaction between Gα_i_ and AC5 by using the FRET-based assay (20). Consistent with the previous study (20), treatment of the cells with clonidine decreased ΔF_CFP_ and increased ΔF_YFP_, indicating that Gα_i1_ interacted with AC5. These effects of clonidine were abolished in cells treated with DAT but not with DAT_S571A_ (Fig. 5*E*). These data indicate that DAT inhibits the interaction of Gα_i_ with AC5 through the demyristoylation of Gα_i_, resulting in abrogation of the Gα_i_-dependent signal transduction.

The article "DAT (deacylating autotransporter toxin) from Bordetella parapertussis demyristoylates Gαi GTPases and contributes to cough" was retracted in 2025. Reasons: fabricated or falsified data; an official misconduct investigation; misconduct by an author; unreliable results or conclusions.

### DAT Vaccination Prevents *B. parapertussis*–Induced Coughing.

Previous studies reported that acellular pertussis vaccines containing pertussis toxoid prevented *B. pertussis*–induced coughing, but not bacterial colonization, in humans and experimental animal models (31, 32). Our results demonstrate that DAT contributes to cough production in *B. parapertussis* infection in place of PTx in *B. pertussis* infection. Indeed, neither the bacterial inoculation of Δ*dat* nor of *dat*_S571A_ caused coughing, while both strains showed equivalent colonization in mouse respiratory organs (Fig. 6 *A* and *B*), indicating that DAT contributes to cough production but not bacterial colonization. These results prompted us to examine whether immunization with DAT prevents *B. parapertussis*–induced coughing. Mice immunized with the diphtheria-pertussis-tetanus-inactivated polio vaccine (DPT-IPV), which is currently used as an acellular pertussis vaccine in Japan, exhibited reduced levels of cough production in response to the inoculation of *B. pertussis*, but not *B. parapertussis*, which is consistent with previous observations (31–33). Meanwhile, immunization with DAT, which was inactivated by formalin treatment, or DAT_S571A_ protected mice from coughing after the inoculation of *B. parapertussis*, but not *B. pertussis*, regardless of the bacterial colonization levels (Fig. 6 *C* and *D*). These results indicate that DAT has potential as a vaccine antigen to prevent *B. parapertussis*–induced coughing.

**Fig. 6.** Protective effects of immunization with DAT against *B. parapertussis*–induced coughing. (*A* and *B*) Cough production in mice inoculated with *B. parapertussis* (Bpp) 12822. The sum of coughs from days 4 to 14 postinoculation is shown (*A*). SS medium without bacteria was used for mock inoculation. The number of bacteria recovered from the tracheas and lungs was counted on day 14 (*B*). (*C* and *D*) Cough production in immunized mice after bacterial inoculation. Mice that had been immunized twice with the DPT-IPV, formalin-inactivated DAT, DAT_S571A_, and/or aluminum hydroxide (Alum) were inoculated with *B. pertussis* (Bp) 18323 (5 × 10^6^ colony forming units (CFU)) or *B. parapertussis* 12822 (5 × 10^7^ CFU). The sum of coughs from days 4 to 14 postinoculation is shown (*C*). The number of bacteria recovered from the tracheas and lungs was counted on day 14 postinoculation of the bacteria (*D*). Each horizontal bar represents the mean and SEM (*A* and *C*, n = 8) or the geometric mean and geometric SD (*B* and *D*, n = 8). Data were obtained from two independent experiments and statistically analyzed by one-way ANOVA with Tukey’s multiple-comparison test (*A* and *C*) or the Kruskal–Wallis test with Dunn’s multiple-comparison test (*B* and *D*). ****P < 0.0001.

The article "DAT (deacylating autotransporter toxin) from Bordetella parapertussis demyristoylates Gαi GTPases and contributes to cough" was retracted in 2025. Reasons: fabricated or falsified data; an official misconduct investigation; misconduct by an author; unreliable results or conclusions.

## Discussion

*B. parapertussis* detected in patients with pertussis-like symptoms was considered the cause of patients’ coughing (1, 2), although no experimental evidence supported this assumption. In this study using the mouse model, we first demonstrated that *B. parapertussis* infection causes host to cough, and *B. parapertussis* DAT, a toxin, was identified as a causative agent to evoke coughing in combination with Vag8 and LPS. Previously, we reported that *B. pertussis* induces host coughing through the cooperative action of PTx, Vag8, and LOS (lipid A) (4). In that mechanism, LOS and Vag8 stimulate and enhance Bdk biogenesis, respectively. Accumulated Bdk stimulates B2R, which transduces stimulatory and inhibitory signals to TRPV1 through Gα_q_ and Gα_s_ GTPases and Gα_i_ GTPases, respectively (*SI Appendix*, Fig. S2). PTx ADP-ribosylates Gα_i_, uncouples it from GPCR (B2R), and interrupts only the Gα_i_-dependent inhibitory signal. As a result, TRPV1 is highly sensitized to evoke coughing. The present study indicates that *B. parapertussis* causes coughing in a similar fashion to *B. pertussis* by utilizing DAT instead of PTx. Unlike PTx, DAT demyristoylates Gα_i_. The myristoyl group attached to Gα_i_ is essential for interaction with the downstream effector AC (26, 27). Therefore, the demyristoylation of Gα_i_ by DAT interrupts Gα_i_-dependent signaling and hypersensitizes TRPV1 to evoke coughing.

The α subunits of heterotrimeric GTPases serve as targets for some bacterial toxins (34). PTx ADP-ribosylates and inactivates Gα_i_. Cholera toxin and *E. coli* heat-labile toxin activate Gα_s_ through ADP-ribosylation. Gα_q_ is targeted by *Pasteurella multocida* toxin and *Yersinia* YpkA: The former activates Gα_q_ by deamidation while the latter inactivates Gα_q_ by phosphorylation. In the present study, we showed that DAT has the unique activity to demyristoylate and inactivate Gα_i_. The GDSL lipase motif present on DAT is shared by several bacterial factors, including *Aeromonas salmonicida* GcaT, *Legionella pneumophila* PlaA, *E. coli* TesA, *Salmonella enterica* serovar Typhimurium SseJ, *Serratia liquefaciens* EstA, *Vibrio parahaemolyticus* hemolysin, and more (16, 17, 35). While the catalytic triads of these bacterial factors, consisting of Ser-His-Asp/Glu, were predicted from the similarity of the amino acid sequences, catalytic key residues of DAT other than Ser remain to be predicted on the basis of the amino acid sequence, suggesting a unique structure of this toxin. In addition, DAT should comprise several domains with distinct functions for cell binding, translocation into the cytoplasm, and enzyme action. DAT also has an aspect as an autotransporter, which is autonomously secreted through its own β-barrel translocator domain. The passenger domains of many classical autotransporters exhibit elongated β helical structures, which may be related to the capability of autonomous secretion (36). Indeed, the AlphaFold2 program predicted structures of the DAT passenger domain consisting of elongated β helices, in which no catalytic triad-like structure was found near the GDSL motif with a catalytic residue Ser571 (*SI Appendix*, Fig. S5), indicating that the conformation of DAT domains alters during the intoxication procedures, or that the predicted structures was incorrect. How the functional domains of DAT are folded into the constrained structure as an autotransporter is for future study. *E. coli* plasmid-encoded toxin (Pet) is a typical example of an autotransporter with the ability to enter target cells and modify intracellular targets (37, 38). The crystal structure of Pet has already been determined, showing the N-terminal extra-domain, and two small domains, which are associated with each other, in addition to the β-helical domain (39). It is worth further investigation to compare the structure of Pet with that of DAT, which we are now trying to determine.

The article "DAT (deacylating autotransporter toxin) from Bordetella parapertussis demyristoylates Gαi GTPases and contributes to cough" was retracted in 2025. Reasons: fabricated or falsified data; an official misconduct investigation; misconduct by an author; unreliable results or conclusions.

*B. pertussis*, *B. parapertussis*, and *Bordetella bronchiseptica*, which are genetically related, share many virulence factors, and commonly cause coughing in host animals, are often collectively called “classical *Bordetella.*” In the present study, we showed that *B. parapertussis*, using DAT instead of PTx, cause cough in a similar way as *B. pertussis*. Some epidemiologic studies suggested that the pertussis-like disease due to *B. parapertussis* is milder in the severity of symptoms and shorter in duration than pertussis due to *B. pertussis* (2, 40). The difference in the disease manifestation may be explained by the low expression levels of Vag8 in *B. parapertussis*, compared to those of *B. pertussis*. Alternatively, differences in the mechanism of toxic action, effective concentrations, and target-cell specificity between PTx and DAT may affect the severity of the diseases. Considering that *B. bronchiseptica*, which does not produce PTx, also causes characteristic paroxysmal coughing in host animals, including dogs, pigs, and various laboratory animals (40–42), we examined whether *B. bronchiseptica*, which possesses an orthologue gene of *dat* (*bb0450*), produces DAT and evokes the cough reflex through the same mechanism; however, unexpectedly, DAT was not detected in the transcript and protein levels in *B. bronchiseptica* (*SI Appendix*, Fig. S6 *A* and *B*). Consistently, *dat*-deficient mutants of *B. bronchiseptica* caused coughing to the same extent as WT (*SI Appendix*, Fig. S6*C*). These observations suggest that *B. bronchiseptica* may produce another virulence factor corresponding to PTx and DAT or cause coughing in a distinct fashion from *B. pertussis* and *B. parapertussis*.

The article "DAT (deacylating autotransporter toxin) from Bordetella parapertussis demyristoylates Gαi GTPases and contributes to cough" was retracted in 2025. Reasons: fabricated or falsified data; an official misconduct investigation; misconduct by an author; unreliable results or conclusions.

The ADP-ribosylating activity of PTx to interrupt the Gα_i_-dependent signal pathway is shown to be responsible for various symptoms in *B. pertussis* infection besides paroxysmal coughing, including leukocytosis, hypoglycemia, and histamine sensitization (43–48). Because DAT, like PTx, interrupts Gα_i_-dependent signal pathways in target cells, similar symptoms could be seen in patients with *B. parapertussis* infection. Although a previous report rejected the idea of leukocytosis in *B. parapertussis* infection (49), further analyses of the function of DAT, such as toxicity strength, in vivo half-life, and target tissue specificity, may provide insights into differences in the disease manifestation between *B. pertussis* and *B. parapertussis* infections. In addition, comparative studies of DAT and PTx would benefit pertussis prevention. Current acellular pertussis vaccines containing pertussis toxoid show efficacy, especially in preventing paroxysmal coughing in pertussis (31, 32). Meanwhile, some previous reports pointed out that acellular pertussis vaccines did not prevent infection by *B. parapertussis*, which does not produce PTx (50, 51). It is also predicted that acellular pertussis vaccines are ineffective at preventing cough in *B. parapertussis* infection, which our findings confirmed. The present study proposes that DAT is a promising candidate for vaccine antigens against *B. parapertussis*–caused coughing. Indeed, immunization with formalin-inactivated DAT or DAT_S571A_, an enzymatically inactive mutant of DAT, preferentially protected mice from coughing after *B. parapertussis* infection. Considering that paroxysmal coughing imposes a serious burden on patients, acellular pertussis vaccines containing DAT could be a bivalent vaccine to prevent pertussis patients from cough production caused by both *B. pertussis* and *B. parapertussis* infections.

## Materials and Methods

*Bacterial Strains, Construction of Plasmids and Mutants, Purification of Recombinant Proteins, LOS and LPS Preparation, Cough Analysis, Vaccination, Measurement of cAMP, Protein Identification by Mass Spectrometry, Deacylase Assay, Click Chemistry, FRET Assay*, and other commonly utilized methods are given in *SI Appendix*. Statistical analyses were performed using Prism 9 (GraphPad Software) as previously reported (52). Data were represented as described previously with slight modifications (52).

The article "DAT (deacylating autotransporter toxin) from Bordetella parapertussis demyristoylates Gαi GTPases and contributes to cough" was retracted in 2025. Reasons: fabricated or falsified data; an official misconduct investigation; misconduct by an author; unreliable results or conclusions.

## Supplementary Material

Appendix 01 (PDF)

Movie S1. A mouse 9 days after inoculation with *B. parapertussis* 12822.

Movie S2. A mouse 9 days after inoculation with SS medium.

## Data Availability

All study data are included in the article and/or supporting information. Data deposited in publicly accessible databases are not included in the article.
